# Detection of Heart Arrhythmia on Electrocardiogram using Artificial Neural Networks

**DOI:** 10.1155/2022/1094830

**Published:** 2022-08-05

**Authors:** Malek Badr, Shaha Al-Otaibi, Nazik Alturki, Tanvir Abir

**Affiliations:** ^1^The University of Mashreq, Research Center, Baghdad, Iraq; ^2^Department of Medical Instruments Engineering Techniques, Al-Farahidi University, Baghdad 10021, Iraq; ^3^Department of Information Systems, College of Computer and Information Sciences, Princess Nourah bint Abdulrahman University, P. O. Box 84428, Riyadh 11671, Saudi Arabia; ^4^Department of Business Administration, Faculty of Business and Entrepreneurship, Daffodil International University, Dhaka, Bangladesh

## Abstract

The electrocardiogram, also known as an electrocardiogram (ECG), is considered to be one of the most significant sources of data regarding the structure and function of the heart. In order to obtain an electrocardiogram, the contractions and relaxations of the heart are first captured in the proper recording medium. Due to the fact that irregularities in the functioning of the heart are reflected in the ECG indications, it is possible to use these indications to diagnose cardiac issues. Arrhythmia is the medical term for the abnormalities that might occur in the regular functioning of the heart (rhythm disorder). Environmental and genetic variables can both play a role in the development of arrhythmias. Arrhythmias are reflected on the ECG sign, which depicts the same region regardless of where in the heart they occur; thus, they may be seen in ECG signals. This is how arrhythmias can be detected. Due to the time limits of this study, the ECG signals of individuals who were healthy, as well as those who suffered from arrhythmias were divided into 10-minute segments. The arithmetic mean approach is one of the fundamental statistical factors. It is used to construct the feature vectors of each received wave and interval, and these vectors offer information regarding arrhythmias in accordance with the agreed-upon temporal restrictions. In order to identify the heart arrhythmias, the obtained feature vectors are fed into a classifier that is based on a multilayer perceptron neural network. In conclusion, ROC analysis and contrast matrix are utilised in order to evaluate the overall correct classification result produced by the ECG-based classifier. Because of this, it has been demonstrated that the method that was recommended has high classification accuracy when attempting to diagnose arrhythmia based on ECG indications. This research makes use of a variety of diagnostic terminologies, including ECG signal, multilayer perceptron neural network, signal processing, disease diagnosis, and arrhythmia diagnosis.

## 1. Introduction

The heart, one of the most sensitive organs of the human body, has a critical role in the functioning of the body. The heart is responsible for pumping the blood necessary for the functioning of tissues and organs. When we look at our circulatory system, there are two types of circulation. These are the small circulation and the large circulation. The small circulation carries low-oxygen blood to the lungs and returns it to the heart after the blood's oxygen content is increased. The great circulation carries blood from the heart to other parts of the body. Although it is a closed system in both circuits, it starts and ends in the heart. The heart consists of three layers, from the outer part to the inner part, as Pericardium, Myocardium, and Endocardium [1]. The muscles in the myocardium, which makes up most of the heart's weight, are the layer where contractions take place. The muscle cells of the myocardium are in layers and completely surround the blood chambers. When the walls of a blood chamber contract, they contract and pressure is applied to the blood in the chamber. About 1% of the cells in the heart is not involved in contraction and are specialized for stimulating the heart. These cells form a network constituting the heart's conduction system and electrically communicate with the heart muscles through their gap junctions. The heart is rich in sympathetic and parasympathetic nerve fibers. The effects of the autonomic nervous system on the heart are regulating, that is, it increases or slows the heart rate and is not necessary for the formation of heartbeats [2]. The heart, which is the basis of our circulatory system, due to its function, the slightest malfunction in its functioning affects the whole body negatively. Disorders in the functioning of the heart are generally called Arrhythmia (Rhythmia Disorder) [3]. The arrhythmia word meaning is the absence of rhythm, but it is used in the sense of deviation from the sinus rhythm, which is called a healthy rhythm. It can be defined as a rhythm arrhythmia caused by the formation of normal or abnormal stimuli, the transmission of abnormal stimuli, or a combination of both. Arrhythmias can be grouped into four main classes: sinus node abnormalities, supraventricular arrhythmias, ventricular arrhythmias, and blocks [4]. Rhythm disorders in the heart also form the basis of some circulatory system-based diseases that will directly affect blood pressure. These irregular changes in blood pressure can cause paralysis, stroke, and even death. Rhythm disorders related to heart rate can be examined in two classes in general. These are tachycardia and barycardia. Tachycardias occur when the heart rate is greater than 100 beats per minute. Barycardia is the name given to rhythm disorders observed in cases where the heart rate is less than 60 beats per minute [5]. In general, cardiac arrhythmias are abnormalities or disturbances in the electrical behavior of the heart. These disorders cause arrhythmia in abnormalities in the heart rate and rhythm. Considering the role of the heart on the circulatory system, the time between two heartbeats during the blood's arrival and exit from the heart is important for the diagnosis and diagnosis of rhythm disorder. In simpler terms, the duration of contraction and relaxation of the heart should be close to each other in people who do not have a rhythm disorder. The absence of periodic intervals or the fact that the start and end times are longer or shorter than certain values are signs of arrhythmia [6]. In ECG measurements, such arrhythmias manifest spontaneously as deformations or irregularities in the observed waveform. Rhythm disorders generally occur for three reasons: psychiatric causes, physical and emotional stress-related causes, and cardiac causes [5, 6]. Considering these factors, diagnosis, and classification of rhythm disorders are important for the treatment of the disease.

Artificial neural networks (ANNs) are computer systems that can learn from the features of the nervous system, derive new information using the new information learned, and work similarly to decision-making structure [7, 8]. ANN has emerged as a result of mathematical modeling of the learning process by taking the human brain as an example. It started with the modeling of neurons, which are the biological units that make up the brain, and continued with its application in computer systems, and later on, it became used in many areas depending on the development of computer technologies. These systems, which are inspired by the working principle of the human brain, have many features according to their usage areas.

Some of them can perform machine learning since they consist of many cells, they can perform complex functions by working simultaneously, they can produce meaningful information from the numerical information used during training, they can learn by using examples, they can be used in perception-oriented events, and they have features such as pattern association and classification. Artificial nerve cells are similar in structure to biological nerve cells. Artificial neurons form artificial neural networks by connecting between them just like our real nervous system. An artificial neuron consists of five parts: inputs, weights, summation function, activation function, and outputs. Activation functions are functions that process the input value to the ANN cell and calculate the output that the cell will produce in response to this input. The “Sigmoid function” is generally used as the activation function in the “Multi-layer perceptron” model, which is widely used today. In the study of in the classification of ECG arrhythmias using the Class modular CGY, it was tried to automatically detect arrhythmic signal anomalies that could help in the diagnosis. Multilayer Back Propagation Algorithm (WGY), one of the learning techniques based on neural networks, and Class-Module concept were applied to two ECG datasets. By using the Class-Module concept with class-based feature selection, it is aimed to obtain durable modules that also provide size reduction, and the RELIEF technique is used for this. The performance of learning techniques has been tried to be increased by using feature selection (Decision Trees, SVM-Cyclic Feature Reduction) and feature expansion (Principal Component Analysis) dimension reduction techniques. Decision Trees and Support Vector Machines have been tested on arrhythmia datasets for comparison purposes. WGY gives approximate results with SVM, better than decision trees on both ECG datasets. It has been observed that the classroom-modular WGY, though slightly less successful, has additional advantages over WGY [9].

In our study, ECG signals were divided into segments, waves, and intervals based on temporal boundaries, and the feature vector of each segment was obtained with the help of the arithmetic mean, which is one of the basic statistical parameters. Arrhythmias occurring in the heart were determined by using these obtained feature vectors as an input to the MPNN model. For this purpose, ECG signals are divided into 10-minute segments of equal length. These sections are divided into sub-sections (segments, waves, and intervals) that provide information about arrhythmias according to the temporal limitations accepted for each segment and wave interval, and the arithmetic mean of each interval is used as an input to the MPNN model for arrhythmia detection. As a result, it has been shown that the proposed approach achieves high classification accuracy in detecting arrhythmia from ECG signs.

## 2. Materials and Method

### 2.1. ECG Sign Used

The “physio net ECG databases” database was used as an ECG signal. “MIT-BIH Normal Sinus Rhytm Database” [10] was used for healthy ECG sign and “MIT-BIH Arrhythmia Database” for arrhythmia sign. Normal Sinus database obtained at Boston's Beth Israel Hospital Arrhythmia Laboratories includes 18 long-term ECG recordings. Measured from 5 men aged 26 to 45 and 13 women aged 20–50. The arrhythmia database was randomly selected from over 4000 records measured at Boston's Beth Israel hospital between 2010 and 2015.

#### 2.1.1. Temporal Limits of ECG Signal

The ECG signature is characterized by a repetitive wave sequence of *P*, QRS, and *T* waves associated with each heartbeat. The QRS complex formed by ventricular depolarization and atrial repolarization is the most striking. As soon as the positions of the QRS complexes are found, *P*, *T* waves and QT, ST segments all appear. The locations of other waves of the ECG, such as the ECG, are determined by the position of the QRS complexes. The intervals in the ECG signs have some temporal characteristics [11]:

*P* wave: Normally, the amplitude of the *P* wave is less than 2.5 mm and the width is less than 0.12 s in all leads.
PR interval: In adults, the PR interval of 0.12–0.20 seconds is considered the normal value.
QRS complex: The duration of the *Q* wave is shorter than 0.04 sec and cannot exceed 25% of the total QRS duration. The duration of the QRS complex is a maximum of 0.11 s.
ST segment: ST segment duration varies inversely with the heart rate and ranges from 0 to 0.15 sec.
*T* wave: It shows the repolarization of the ventricles. The duration of the normal *T* wave in adults is 0.10–0.25 sec.
RR interval: It is the distance between two *R* points.
QT interval: The heart rate corrected QT interval is expressed as QTc. QTc is calculated by dividing the QT duration by the square root of the RR duration (Bazett Formula) [12]. The upper limit of the corrected QT interval (QTc_B) calculated according to Bazett's formula is 0.44 sec and is calculated with equation as follows [10]:
  (1) $$\begin{array}{c} \text{QTB }=\;\frac{\text{QT}}{\sqrt{\text{RR}}}. \end{array}$$

Here, QTcB indicates the corrected QT interval calculated using Bazett's formula.

#### 2.1.2. Feature Extraction Based on Calculation of Temporal Intervals from ECG Signals

*(1) R Point Detection with Pan-Tompkins Algorithm*. In this study, arithmetic mean-based feature vectors of *P*, PR, QRS, QT, ST, T, and RR intervals of ECG signals were calculated using the temporal distance from *R* point. Pan-Tompkins algorithm was used to detect the *R* point in the ECG signal. The Pan-Tompkins algorithm consists of five steps: band-pass filter, derivative, squarer, sliding window integration, and threshold adjustment. The first step of the Pan-Tompkins algorithm is to apply a band-pass filter to filter out the noise in the ECG signals. The band-pass filter used in the Pan-Tompkins algorithm is obtained with low-pass and high-pass filters. For the high-pass filter, the sampling frequency is 200 Hz, the cutoff frequency is 11 Hz, and the shift amount is 5 samples, i.e., 25 msec. The cutoff frequency of the high-pass filter is 200 Hz, the sampling frequency is 5 Hz, the shift amount is 16 samples, that is, 80 msec [13].

In the derivation stage, the filtered ECG signal was applied to the derivative receiver to make the QRS clear, and the low-frequency components were suppressed, and the ECG signal free from the low-frequency components was obtained. Finally, the smoothing process is performed with the integration of the squarer and the sliding window. In this study, after the *R* points in the QRS segment were determined, signal groups were formed according to the temporal intervals of the waves in the ECG signal and the averages of the temporal distances to the detected *R* points were calculated.

*(2) Calculation of Temporal Intervals of ECG Signal.*

**Step 1 .**

Deviation in RR intervals: The mean (RRort) of all RR points in the sign is calculated, how much the distance of each RR block differs from the calculated mean. The low difference indicates that the *R* points continue periodically. If the difference is large, it means that the *R* points are not formed at regular time intervals. The mean of the RR interval deviations is calculated by equation below.

(2) $$\begin{array}{c} {\text{RR}}_{\mathrm{deviation}}=\sum_{i=1}^{{\text{RR}}_{\mathrm{End}}}\frac{\left|\text{RRi}-\text{RRort}\right|}{\text{RRnumber}}\;. \end{array}$$

RR_ort_ represents the mean of all RR intervals in the sign, RRnumber represents the number of all RR intervals, and RRdeviation is the mean of the difference of all RR intervals to the calculated RRort value.

**Step 2 .**

QRS interval: The *Q* interval cannot exceed 25% of the total QRS and the total duration of the QRS cannot exceed 0.11 sec. Also, *Q* should be <0.04 sec.

Assuming the *R* point is the middle of the QRS block, QRShalf: 0.11/2 = 0.055.

*Q*: 0.11/4 = 0.0275. (It also complies with condition *Q* < 0.04). *R*_half_: QRS_half_–*Q* then *R*_half_ = 0.055–0.0275 = 0.0275 *R* = 2*R*_half_: 0.055 and S: QRS–S–*R* if *S* = 0.0275.

**Step 3 .**

The temporal distances of the intervals to the point *R*:

The temporal distances of the *P*, PR, *Q*, *S*, *T*, and QT intervals to the *R* point are determined.

- *P*_start_: The temporal distance of the *P* wave origin from the *R* point.
- *P*_bitis_: The distance from the *P* wave end point to the *R* point.
- PR_start_: The temporal distance from the PR interval starts point to the *R* point.
- PR_end_: The temporal distance of the PR interval end point from the *R* point. *Q*_start_: The temporal distance of the *Q* interval start point from the *R* point. Stop: The temporal distance of the S interval end point from the *R* point.
- ST_start_: The temporal distance of the ST segment origin from the *R* point.
- ST_end_: The temporal distance of the ST segment end point to the *R* point. *T*-origin: The temporal distance of the *T*-wave origin from the *R* point. Tend: The temporal distance of the *T* wave end point to the *R* point.
- QTc_start_: the temporal distance from the corrected QT interval start point to the *R* point.
- QTc_end_: The temporal distance of the corrected QT interval endpoint to the *R* point.
- *R*_half_: The *R* wave is half the width in time.

**Step 4 .**

*P* interval: The calculation of the distance of the *P* interval from the *R* point.

- If *P*_start_ = PR + QR then 0.2 + 0.055 = 0.255 sec.
- *P*_end_ = *P*_start_ − 0.10 = 0.155 sec.

**Step 5 .**

PR interval: the intervals in calculating the PR interval are expressed.

- PR_start_ = *P*_start._
- PR_end_ = PR_start_ − 0.2 = 0.055 sec.

**Step 6 .**

QRS interval: *Q*_start_ = 0.55 sec

Stop = 0.55 sec.

**Step 7 .**

ST segment length: the intervals in calculating the length of the ST segment.

- ST_start_ = Stop.
- If ST_end_ = ST_start_ + 0.15.
- ST_end_ = 0.205 sec.

**Step 8 .**

*T* interval: the intervals in the calculation of the *T* wave.

- *T*_start_ = ST_end._
- If *T*_end_ = *T*_start_ + 0.25 then Tend = 0.455 sec.

**Step 9 .**

QTc interval: the QTc interval is calculated according to Bazett's formula.

- QTcstart = *Q*_start._
- QTcfinish = QTc − *R*_half._

The averages of all waves and intervals were calculated according to the steps shown above as an example. In the calculation, 90 arrhythmias and 90 normal sinus rhythms, a total of 180 sign segments were used.

### 2.2. Artificial Neural Network Model

Who studied how the brain learns, laid the foundations of today's neural network theory. He studied the relations of nerve cells with each other and developed the neural network theory on this basis. Although it is not known exactly how the brain works, this model, which has been developed, does not fully show the learning structure of the brain. However, there are many neural network models with success rates of 99%. Artificial neural network (ANN) is a model that tries to transfer the layered and parallel structure of the human brain's nerve cells to the digital environment, and it comes together from more than one nerve cell, just like the human nervous system. Biological and artificial nerve cells are seen in Figure 1 [14]. ANN has both hardware and software models, but the inflexibility of hardware models have highlighted the use of software models.

The biological nerve cell generally consists of four parts:

- Dendrite: its function is to transmit signals transmitted from other nerve cells to the nucleus of the nerve cell.
- Soma: it is the centre that collects all transmitted signals.
- Axon: it is responsible for transmitting the information it receives to the next nerve cell nucleus.
- Synapsis: after processing the total information from the axon, it transmits it to the dendrites of other nerve cells.

As seen in Figure 1 (b), in the artificial neuron, *X* carries the input signals and W carries the weight coefficient of that signal. A weighted sum of all input signals is obtained in the kernel. All these total sign is denoted by Yin. Yin is sent to the synapse as an input to the thresholding function. The result produced by the thresholding function in the synapse is expressed as *Y* and directed to enter the other cell.

Like the real nervous system, ANN can perform operations such as learning, memorizing, and revealing the relationship between data. It transfers the data from the dendrites to the synapses by passing them through threshold functions. There are three types of threshold functions commonly used in ANN models [15]:

- Hard limiter function
- Threshold function
- Sigmoid function.

#### 2.2.1. Arrhythmia Detection with Multilayer Neural Network

Artificial neural networks can be single-layered or multi-layered, depending on their intended use. Interlayers used in multi-layer networks can increase the capability of the network and negatively affect the uptime [16–19]. Multilayer networks are divided into layers as input layer, middle layer, and output layer. The input layer takes the input values coming from the outside to the neural network and directs them to the middleware. There is no information processing in this layer. As there may be more than one input, each incoming input information is sent directly to the next layer. Each processing element in the input layer depends on the elements in the next layer. The middle layers process the input information from the input layer, which is the upper layer, and send the outputs to the next layer. There may be more than one intermediate layer in a Perceptron Neural network, or it may consist of more than one nerve cell in each layer. Each cell in the middle layer is connected to all other cells in the next layer. The output layer processes the data from the middleware and sends the outputs produced by the network to the neural network outputs. Each element has an output. Multilayer Perceptron Neural (MPN) networks work with the teacher-learning method. Well, both input values and output values corresponding to these inputs are shown to these networks during training. The task of the network is to produce the output corresponding to that input for each given input. It is a generalization of Delta learning rule based on least squares learning as a learning rule. The generalized “Delta rule” consists of two phases: forward calculation and backward calculation. In order for the network to learn, it needs a set of examples called a training set. MPN's working system; collecting samples, determining the topological structure of the network, choosing the learning parameters, entering the initial value of the weights, selecting the samples from the learning set and showing them to the network, making forward calculations during learning, comparing the actual output with the expected output, and changing the weights [20–22]. As seen in Figure 2 7 feature vectors, namely, Port, PR_ort_, QRSort, ST_ort_, *T*_ort_, QT_ort_, and RR_ort_, were used as input values to the MPNN model, which has 10 neurons in the hidden layer, for arrhythmia detection from ECG signals.

The classifier model, whose tangent-hyperbolic activation function was chosen as the activation function, was trained with the Levenberg–Marquardt (LM) back propagation algorithm. The MPNN Classifier model was run 100 times and the final result was calculated by averaging the classification successes obtained. For training, feature vectors of 90 healthy signs and feature vectors of 90 arrhythmia signs were applied to the classifier model.  Table 1 shows sample input values used in MPNN.

The average values obtained from the normal and arrhythmic signs as a result of the calculations are shown in Figure 3.

A 10-piece cross-validation criterion based on random sample selection was used to measure the generalized success of the classifier. In this method, the obtained feature vectors are randomly distributed into three groups as training, validity, and test data. The training data was chosen to contain 70% of all data (126 samples), while the validity and test data included 15% (54 samples) (Table 2). When the success of the model in the validity data reached the highest level, the training was stopped. The classification success of the model was evaluated with the help of statistical criteria.

### 2.3. Evaluation of Results with ROC Analysis

The ROC curve is calculated as the ratio of sensitivity to precision and is used in binary classification systems where the discrimination threshold differs. In simpler terms, ROC can also be defined as the ratio of true positives to false positives. In the ROC curve, the criteria generally used in the evaluation are sensitivity, general accuracy, specificity, positive predictive value, and negative predictive value. By using Figure 4, the limit values of the tests for these criteria can be determined [23–28].

Sensitivity (%): It shows what percentage of people known to have the disease can be diagnosed with the recommended method. The sensitivity formula is given in equation below.
  (3) $$\begin{array}{c} \frac{S_{1}}{S_{1}+S_{3}}=\frac{\text{TP}}{\text{TP}+\text{FN}}. \end{array}$$
Specificity (%) (specificity): It shows what percentage of those who do not have the disease (who are healthy) can be recognized. The specificity formula is given as
  (4) $$\begin{array}{c} \frac{S_{4}}{S_{2}+\text{FP}}=\frac{\text{TN}}{\text{TN}+\text{FP}}. \end{array}$$
Plus, interpretation power (%) (+ predictive value): it indicates how much disease is detected by the positive findings (conformity to the known method). In (5), the plus interpretation power formula is given.
  (5) $$\begin{array}{c} \frac{S_{1}}{S_{1}+S_{2}}=\frac{\text{TP}}{\text{TP}+\text{FP}}. \end{array}$$
Negative power of interpretation (%) (– predictive value): it indicates how much the negative findings indicate the absence of disease. The negative interpretation power formula is given as.
  (6) $$\begin{array}{c} \frac{S_{4}}{S_{3}+S_{1}}=\frac{\text{TN}}{\text{TN}+\text{FN }}. \end{array}$$
General accuracy (%) (accuracy): it shows what percentage of sick and healthy people can be recognized. The general accuracy formula is given as
  (7) $$\begin{array}{c} \frac{S_{1}+S_{4}}{S_{1}+S_{2}+S_{3}+S_{4}}=\frac{\text{TP}+\text{TN}}{\text{TP}+\text{TN}+\text{FP}+\text{FN}}. \end{array}$$

Statistical criteria were used on the final correct classification success test data of the MPNN model we used. The most basic criteria for this assessment are specificity, sensitivity, and overall classification accuracy.

Confusion matrix and ROC curve analysis are used in order to evaluate success in case the distribution of sample data on the basis of class is very different and success is high [29–34]. The confusion matrix obtained as a result of the proposed model's classification of ECG signals is shown in Figure 3.

As it can be seen from Figure 3, although misclassification is not made for the diagnosis of arrhythmia in the proposed approach, misclassification can be made for a healthy individual without arrhythmia, albeit very low. Using equations (3)–(5), a specificity rate of 93.3%, a sensitivity rate of 100%, and a TDS rate of 96.3% were calculated. This shows that the classifier has high success rates. Figure 4 shows the ROC analysis curve of the classification experiment performed to diagnose arrhythmia from ECG signals.

Based on the ROC curve analysis as shown in Figures 4 and 5 the proposed approach has acceptable classification capability in diagnosing arrhythmia. Accordingly, large areas under the ROC curves indicate that it is a classifier model with high specificity and sensitivity.

## 3. Results and Discussion

For arrhythmia detection in ECG signals, high classification success rates have been achieved when feature vectors obtained with the help of an arithmetic mean from signals segmented into temporal segments and waves are used as an input to a MPNN model. Since the lengths of the signals are different in the data sets used, the signals were divided into equal-length pieces before processing. In addition to the intervals used in the arrhythmia diagnosis studies in the literature, all wave segments and intervals formed during the contraction and relaxation of the heart were used as inputs in MPNN. It has been shown that the segment and wave intervals of the 10-minute segments of the ECG signals are important feature vector in arrhythmia detection. The obtained results were evaluated using ROC analysis, and as a result, it was seen that high classification accuracy rates were obtained by applying the statistical properties of the wave intervals of the segmented ECG signals to an ANN-based classifier model. It is an important finding that an ANN model using the temporal limits of segment waves and intervals of ECG signals achieves high success in detecting arrhythmia. In future studies, a system that can diagnose arrhythmias according to the given criteria, can select among arrhythmia types, can be developed, and specialized arrhythmia detection can be carried out. Segment waves and intervals in the heart can be used to classify arrhythmias. The expert system model can be added to the artificial intelligence model currently used. With the hybrid system obtained, a model can be created that can learn and decide on itself for the diagnosis of the disease, learn the past signs, and detect possible symptoms that may develop in the future. Our study can be arranged to be integrated into mobile devices, and a tracking system can be developed for the use in the health sector and in daily life. In this way, a system that can instantly learn the conditions of critical patients and make decisions without losing time for intervention can be obtained and early intervention can be provided. It is possible to use these systems, which are mentioned in future studies, not only during the diagnosis of the disease, but also during the use of drugs and treatment.

## 4. Conclusion

The classification performance of various feature sets used in ECG signal separation can vary. As a result, the Pan-Tompkins algorithm is recommended in this study for selecting the appropriate feature set for the signal. The selection pool was made up of features extracted from different wavelet types. The results also showed that the genetic algorithm method can detect features that improve classification accuracy, and that the feature set derived from coefficients selected at various levels of different types of wavelets improves ECG arrhythmia classification performance when compared to the coefficients derived from the standard uniform wavelet. In future research, it is hoped to test more parameters in order to improve the Pan-Tompkins algorithm's performance by including features obtained from various methods in the feature selection set.

## Figures and Tables

**Figure 1:** (a) Biological nerve cell structure and (b) artificial neuron structure.

**Figure 2:** Multilayer perceptron neural network (MPNN) class model.

**Figure 3:** Average values obtained from normal and arrhythmic signs ((a) *P*_ort_ values; (b) PR_ort_ values; (c) QRS_ort_; (d) ST_ort_; (e) *T*_ort_ values; (f) QT_ort,_ and RR_ort_ values obtained from healthy and arrhythmia signals).

**Figure 4:** Confusion matrix for arrhythmia diagnosis.

**Figure 5:** ROC analysis curve of classification.

**Table 1:** Example input values used in MPNN.

−0.32439	−0.31479	0.047868	−0.23542	−0.40862	−0.27346	0.027801	1	0
−0.31515	−0.30804	0.073892	−0.23052	−0.38382	−0.26372	0.423111	1	0
−0.31038	−0.30561	0.068777	−0.22866	−0.38145	−0.26014	0.421215	1	0
−0.30523	−0.33142	0.012525	−0.17322	−0.39915	−0.10686	0.030321	1	0
−0.29537	−0.32213	0.00847	−0.19931	−0.39377	−0.18664	0.446077	1	0
−0.29879	−0.31608	−0.0471	−0.20281	−0.38134	−0.18024	0.451827	1	0
−0.22591	−0.23854	0.200567	−0.21593	−0.48883	−0.25299	0.033917	1	0
−0.24436	−0.25376	0.137639	−0.22789	−0.46865	−0.24487	0.363481	1	0
−0.22831	−0.24922	0.07375	−0.22680	−0.46672	−0.22632	0.317504	1	0
−0.26414	−0.21274	0.107591	−0.07347	−0.36917	0.07149	0.131064	1	0
−0.14564	−0.13468	0.333994	−0.03551	−0.22433	−0.11605	0.054218	0	1
−0.13861	−0.12987	0.378555	−0.02868	−0.20941	−0.08673	0.392148	0	1
−0.13971	−0.13435	0.383486	−0.04665	−0.18899	−0.13101	0.354666	0	1
−0.1408	−0.13496	0.380989	−0.04530	−0.18077	−0.13068	0.359025	0	1
−0.14555	−0.13962	0.395855	−0.04032	−0.1741	−0.13047	0.368294	0	1
−0.17153	−0.1633	0.418286	−0.03743	−0.14792	−0.14097	0.375346	0	1
−0.16082	−0.15058	0.368256	−0.02273	−0.16884	−0.09294	0.325423	0	1
−0.1637	−0.15382	0.382274	−0.02667	−0.15914	−0.10595	0.363618	0	1
−0.16178	−0.15104	0.37407	−0.0304	−0.16452	−0.10913	0.357767	0	1
−0.16122	−0.15004	0.395915	−0.03601	−0.15363	−0.13164	0.399601	0	1

**Table 2:** Criteria used in the evaluation of diagnostic and screening tests.

Test result	Arrhythmia patient	Healthy samples	Total
	(Positive)	(Negative)	
Test (+)	*S *_1_(TP)	*S *_2_ (FP)	*S *_1_ + *S*_2_
Test (−)	*S *_3_ (FN)	*S *_3_ (TN)	*S *_3_ + *S*_4_
Total	*S *_1_ + *S*_3_	*S *_2_ + *S*_4_	*S *_1_ + *S*_2_ + *S*_3_ + *S*_4_
TP : True positive; FP : False positive; FN : False negative; TN : True negative.			

## Data Availability

The data used to support the findings of this study are included within the article.

## References

[1] Gálfiová P., Polák Š., Mikušová R. (2017). The three-dimensional fine structure of the human heart: a scanning electron microscopic atlas for research and education. *Biologia*.

[2] Muhammad B. A. M. (2022). The role of universities in developing societies by accreditation on scientific research. *Scientific Journal Al-Imam University College*.

[3] van Bilsen M., Patel H., Bauersachs J., Böhm M., Borggrefe M. (2017). The autonomic nervous system as a therapeutic target in heart failure: a scientific position statement from the Translational Research Committee of the Heart Failure Association of the European Society of Cardiology: autonomic nervous system therapy in HF. *European Journal of Heart Failure*.

[4] Tse G. (2015). Mechanisms of cardiac arrhythmias. *Journal of Arrhythmia*.

[5] Gaztañaga L., Marchlinski F., Betensky B. (2011). Mechanisms of cardiac arrhythmias. *Revista Española de Cardiología*.

[6] Alazzam M. B., Tayyib N., Alshawwa S. Z., Ahmed M. (2022). Nursing care systematization with case-based reasoning and artificial intelligence. *Journal of Healthcare Engineering*.

[7] Abdelmoneem S., Said H., Saad A. (2020). Arrhythmia disease classification and mobile based system design. *Journal of Physics: Conference Series*.

[8] Verheyen T., Decloedt A., Clercq D., deprez P., Sys S. U., van Loon G. (2010). Electrocardiography in horses-Part 2: how to read the equine ECG. *Vlaams Diergeneeskundig Tijdschrift*.

[9] Abdullah Hamad A., Thivagar M. L., Bader Alazzam M., Alassery F., Hajjej F., Shihab A. A. (2022). Applying dynamic systems to social media by using controlling stability. *Computational Intelligence and Neuroscience*.

[10] Grossi E., Buscema M. (2008). Introduction to artificial neural networks. *European Journal of Gastroenterology and Hepatology*.

[11] Amjad A., Abdel Rahim Al-B. (2022). The possibility of implementing industrial incubators and their role in the development of small industry and medium in Iraq. *Scientific Journal Al-Imam University College*.

[12] Lee D.-H., Kim Y.-T., Lee S.-R. (2020). Shallow landslide susceptibility models based on artificial neural networks considering the factor selection method and various non-linear activation functions. *Remote Sensing*.

[13] Xu S., Mak M.-W., Cheung C.-C. Deep Neural Networks versus Support Vector Machines for ECG Arrhythmia Classification.

[14] Alazzam M. B., Al-Radaideh A. T., Alhamarnah R. A., Alassery F., Hajjej F., Halasa A. (2021). A survey research on the willingness of gynecologists to employ mobile health applications. *Computational Intelligence and Neuroscience*.

[15] Sharma J., Kumar V., Ayub S., Saini J. (2012). Uniform sampling of ECG waveform of MIT-BIH normal sinus rhythm database at desired intervals. *International Journal of Computer Application*.

[16] Fadhil Jwaid M. (2022). An efficient technique for image forgery detection using local binary pattern (hessian and center symmetric) and transformation method. *Scientific Journal Al-Imam University College*.

[17] Bader Alazzam M., Mansour H., Hammam M. M. (2021). Machine learning of medical applications involving complicated proteins and genetic measurements. *Computational Intelligence and Neuroscience*.

[18] Mondal S., Choudhary P. Detection of normal and abnormal ECG signal using ANN: selected revised papers from the joint.

[19] Dahlberg P., Diamant U.-B., Gilljam T., Rydberg A. (2020). QT correction using Bazett’s formula remains preferable in long QT syndrome type 1 and 2. *Annals of Noninvasive Electrocardiology*.

[20] Pooyan M., Akhoondi F. (2016). Providing an efficient algorithm for finding R peaks in ECG signals and detecting ventricular abnormalities with morphological features. *Journal of Medical Signals and Sensors*.

[21] Ishaq Yousef Al-A., Abdul R. S. (2022). Social intelligence and its relationship to decision quality. *Scientific Journal Al-Imam University College*.

[22] Al-Obeidi A. S., Sultan N. A., Obaid A. R. (2021). The degree of applying electronic learning in the Gifted School/Nineveh in Iraq and what management provided to the students and its relationship to qualitative education under coronavirus (COVID-19) pandemic. *International Journal of Computer Applications in Technology*.

[23] Rasmi M., Alazzam M. B., Alsmadi M. K., Almarashdeh I. A., Alkhasawneh R. A., Alsmadi S. (2020). Healthcare professionals’ acceptance Electronic Health Records system: critical literature review (Jordan case study). *International Journal of Healthcare Management*.

[24] Werbos P. (2009). Intelligence in the brain: a theory of how it works and how to build it. *Neural Networks*.

[25] An H., Ehsan Md A., Zhou Z., Yi Y. Electrical Modeling and Analysis of 3D Synaptic Array Using Vertical RRAM Structure.

[26] Zupan J. (1994). Introduction to artificial neural network (ANN) methods: what they are and how to use them. *Acta Chimica Slovenica*.

[27] Kumar G. (2019). Arrhythmia Detection in ECG Signals Using a Multilayer Perceptron Network. http://ceur-ws.org/Vol-2563/aics_33.pdf.

[28] Enbeyle W., Al-Obeidi A. S. (2022). Trend analysis and prediction on water consumption in southwestern Ethiopia. *Journal of Nanomaterials*.

[29] Işın A., Özdalili S. (2017). Cardiac arrhythmia detection using deep learning. *Procedia Computer Science*.

[30] Kornej J., Schumacher K., Zeynalova S. (2019). Time-dependent prediction of arrhythmia recurrences during long-term follow-up in patients undergoing catheter ablation of atrial fibrillation: the Leipzig Heart Center AF Ablation Registry. *Scientific Reports*.

[31] Hammoudi K., Benhabiles H., Melkemi M. (2021). Deep learning on chest X-ray images to detect and evaluate pneumonia cases at the era of COVID-19. *Journal of Medical Systems*.

[32] Soric M., Pongrac D., Inza I. Using Convolutional Neural Network for Chest X-ray Image Classification.

[33] Latheesh M., Gnana S., Puppala N., Kanmani P. (2021). Chest diseases prediction from X-ray images using CNN models: a study. *International Journal of Advanced Computer Science and Applications*.

[34] Stirenko S., Kochura Y., Alienin O. (2018). Chest X-Ray Analysis of Tuberculosis by Deep Learning with Segmentation and Augmentation. https://arxiv.org/abs/1803.01199.

